# JNK Contributes to the Tumorigenic Potential of Human Cholangiocarcinoma Cells through the mTOR Pathway Regulated GRP78 Induction

This article has been retracted.

**DOI:** 10.1371/journal.pone.0090388

**Published:** 2014-02-28

**Authors:** Chunhong Feng, Kai He, Chunyan Zhang, Song Su, Bo Li, Yuxiao Li, Chun-Yan Duan, Shaokun Chen, Run Chen, Youping Liu, Hong Li, Mei Wei, Xianming Xia, Rongyang Dai

**Affiliations:** 1 Department of Hepatobiliary Surgery of the Affiliated Hospital, Luzhou Medical College, Luzhou, Sichuan, China; 2 Department of Biochemistry and Molecular Biology, Luzhou Medical College, Luzhou, Sichuan, China; 3 Department of Public Health, Luzhou Medical College, Luzhou, Sichuan, China; 4 Affiliated Hospital of Chinese Traditional Medicine, Luzhou Medical College, Luzhou, Sichuan, China; Florida International University, United States of America

## Abstract

Less is known about the roles of c-Jun N-terminal kinase (JNK) in cholangiocarcinoma (CCA). Here, we report that JNK exerts its oncogenic action in human CCA cells, partially due to the mammalian target of rapamycin (mTOR) pathway regulated glucose-regulated protein 78 (GRP78) induction. In human CCA cells, the phosphorylation of eukaryotic initiation factor alpha (eIF2α) results in the accumulation of activating transcription factor 4 (ATF4) and GRP78 independent of unfolded protein response (UPR). Suppression of GRP78 expression decreases the proliferation and invasion of human CCA cells. It's notable that mTOR is required for eIF2α phosphorylation-induced ATF4 and GRP78 expression. Importantly, JNK promotes eIF2α/ATF4-mediated GRP78 induction through regulating the activity of mTOR. Thus, our study implicates JNK/mTOR signaling plays an important role in cholangiocarcinogenesis, partially through promoting the eIF2α/ATF4/GRP78 pathway.

## Introduction

Cholangiocarcinoma (CCA) is a malignancy that arises from the malignant transformation of the epithelial cells of the intrahepatic or extrahepatic bile ducts. CCA has very poor prognosis and is extremely aggressive with restricted treatment options [1], [2], [3], [4]. CCA often arises from background conditions that cause long-term bile duct inflammation, chronic bile duct injury and reparative biliary epithelial cell proliferation [1], [2], [3], [5], [6], [7], [8]. The pathogenesis of CCA is poorly understood. It is known that inhibition the proliferation and invasion of malignant biliary epithelial cells is a potential strategy for the treatment of CCA. In fact, little is known about the molecular mechanism controlling the proliferation and invasion of CCA cells. Elucidation of intracellular proliferation and invasion events is very important in that it will contribute to the development of potential therapeutic strategy for the treatment of CCA.

Glucose-regulated protein 78 (GRP78) is an essential regulator of endoplasmic reticulum (ER) homeostasis due to its essential roles in protein folding and calcium homeostasis regulating [9], [10], [11], [12], [13], [14]. Recent studies have firmly established the role of GRP78 in the development and progression of cancer [15], [16], [17], [18], [19], [20]. GRP78 is induced in a wide variety of cancer cells and cancer biopsy tissues. Recent progress establishes that GRP78 is preferably required for cancer cell survival under pathologic conditions [17], [20], [21], [22]. GRP78 is a promising target for treatment of cancer. However, whether GRP78 is involved in human CCA remains to be elucidated.

c-Jun N-terminal kinases (JNK), an evolutionarily conserved mitogen-activated protein kinase (MAPK), plays an important role in converting extracellular stimuli into a wide range of cellular responses, including inflammatory response, stress response, differentiation, and survival [23], [24], [25], [26], [27], [28], [29], [30], [31]. JNK can suppress the progress of cancer by negative regulation of cell cycle, and by induction of cancer cells apoptosis [32], [33], [34], [35]. JNK also exerts its oncogenic action through promoting inflammation, proliferation, invasion, and angiogenesis [32], [36], [37]. A recent report indicates that inhibiting JNK enhances TGF-β-induced apoptosis of CCA cells, which suggests the link between JNK and CCA [38]. At present, little is known about the role and mechanism of JNK in cholangiocarcinogenesis. Thus, it is necessary to uncover the function of JNK in CCA.

In the present study, we aimed to explore the function and mechanism of JNK in CCA. We found strong expression of phosphorylated JNK and GRP78 in human CCA cells. Additionally, our data reveal that both JNK and GRP78 are important for the proliferation and invasion of human CCA cells. In human CCA cells, eukaryotic initiation factor-alpha (eIF2α)/activating transcription factor 4 (ATF4) signaling contributes to the accumulation of GRP78. Interestingly, JNK maintains high expression of GRP78 through promoting the activation of the mammalian target of rapamycin (mTOR) pathway. Taken together, our findings suggest that GRP78 contributes to the pro-tumorigenic function of JNK in human CCA cells.

## Materials and Methods

### Ethics statement

Human tissues were obtained from the Affiliated Hospital of Luzhou Medical College. This study has been approved by the Luzhou Medical College Ethical Committee. The approval for the use of these specimens with a waiver of consent was granted by the Luzhou Medical College Institutional Review Board.

### Chemicals and antibodies

JNK inhibitor SP600125 (SP), eIF2α phosphatase enzymes inhibitor salubrinal (Sal) and mTOR inhibitor rapamycin (Rap) were purchased from Tocris Bioscience (Bristol, UK). p70S6K inhibitor PF-4708671 (PF) was purchased from Selleck Chemicals (Houston, TX, USA). AP-1 inhibitor curcumin, cell counting kit-8 (CCK8) and ER stress inducer tunicamycin (Tun) were purchased from Sigma (Lyon, France). The eIF4E/eIF4G interaction inhibitor 4EGI-1, mTOR siRNA, GFP siRNA, JNK siRNA, GRP78 siRNA, ATF4 siRNA and antibodies against GRP78, eIF2α and β-actin were purchased from Santa Cruz Biotechnology (Heidelberg, Germany). Antibodies against phospho-eIF2α (Ser-51), phospho-p70S6K (Thr-389), phospho-mTOR (Ser-2448), phospho-Raptor (Ser-863), phospho-c-Jun (Ser-73), phospho-JNK (Thr-183/Tyr-185), phospho-4E-BP1 (Thr-37/46), p70S6K, mTOR, Raptor, c-Jun, JNK, 4E-BP1 and ATF4 were purchased from Cell Signaling Technology (Danvers, MA, USA).

### Cell culture and treatments

Human CCA cell lines QBC939, RBE and HCCC-9810 and hepatocellular carcinoma cell line HepG2 were obtained from ATCC. QBC939, RBE and HCCC-9810 cells were cultured in RPMI-1640 medium, and HepG2 cells were cultured in Dulbecco's modified Eagle's medium supplemented with 10% fetal bovine serum and 1% penicillin/streptomycin in a humidified incubator containing 5% CO_2_ and 95% ambient air at 37°C. The protocol used for GRP78, JNK, ATF4 and mTOR knockdown has been previously described [39].

### Western blot analysis

Cells were lysed in Triton lysis buffer (20 mM Tris, pH 7.4, 137 mM NaCl, 10% glycerol, 1% Triton X-100, 2 mM EDTA, 1 mM PMSF, 10 mM sodium fluoride, 5 mg/ml of aprotinin, 20 mM leupeptin, and 1 mM sodium orthovanadate) and centrifuged at 12,000 g for 15 minutes. Protein concentrations were measured using the BCA assay. Protein samples were denatured with 4×SDS-loading buffer (200 mM Tris, pH 6.8, 8% SDS, 400 mM DTT, 0.4% bromphenol blue, 40% glycerol) at 100°C for 5 minutes and subjected to standard SDS-PAGE and Western blot analysis as previously described [7].

### Cell counting kit-8 assa*y*

Cells were trypsinized and seeded at 3×10^3^ cells/well in 96-well plates. After 24 h, cells were treated with various doses of inhibitors or were transfected with siRNA for indicated time periods. Then, 20 µl of CCK8 solution (5 g/l) in phosphate buffered saline (PBS) was added. After incubated for an additional 2 h, the absorbance value in each well was measured using a microculture plate reader (Bio-Tek, USA) at a wavelength of 490 nm.

### Cell migration and invasion assay

Cells were transferred to 24-well Transwell chambers (Costar, Corning, NY). For migration assay, cells were seeded in the upper Transwell chamber at 1×10^5^ cells/well. For the invasion assay, cells were seeded in the upper Matrigel-coated Transwell chamber at 2×10^5^ cells/well. After incubation at 37°C for indicated time periods, migrated and invaded cells were fixed in 95% ethanol, stained with a solution of 2% crystal violet in 70% ethanol, and counted under an inverted microscope. Three fields were randomly chosen and the numbers of migrated and invaded cells were counted.

### Reverse transcription reaction and real-time PCR

Total RNA was isolated with TRIzol reagent (Invitrogen, Carlsbad, CA, USA) according to the manufacturer's instructions. The reverse transcription reactions were carried out using the M-MLV reverse transcriptase (Promega, Madison, WI, USA) according to the manufacturer's protocol. Results were normalized with 18S. Real-time PCR analyses were performed using SYBR Premix Ex Taq (TaKaRa, Tokyo, Japan). The primers used in this study are as follows: human XBP1 sense primer, 5′-CCT TGT AGT TGA GAA CCA GG-3′ and antisense primer, 5′-GGG GCT TGG TAT ATA TGT GG-3′; human GRP78 sense primer, 5′-ATC ACG CCG TCC TAT GTC GC-3′ and antisense primer, 5′-TCT CCC CCT CCC TCT TAT CC-3′; human ATF4 sense primer, 5′-GTA ACC GAC AAA GAC ACC TT-3′ and antisense primer, 5′-TTT CTC CAA CAT CCA ATC TG-3′; human 18S sense primer, 5′-GGG AGG TAG TGA CGA AAA AT-3′ and anti-sense primer, 5′-ACC AAC AAA ATA GAA CCG CG-3′.

### Statistical analysis

Results were expressed as the mean±SD. Statistical analysis was performed using Student's t test. A *P* value of less than 0.05 was considered statistically significant.

## Results

### JNK promotes the proliferation and invasion of human CCA cells

To investigate the role of JNK in CCA, we first examined the expression of phosphorylated JNK and its downstream target phosphorylated c-Jun in human CCA cells. As shown in Figure 1A, QBC939, RBE and HCCC-9810 cells showed strong expression of phosphorylated JNK and phosphorylated c-Jun. SP600125, a selective inhibitor of JNK, inhibited the phosphorylation of c-Jun in a dose-dependent manner in QBC939, RBE and HCCC-9810 cells (Figure 1B), indicating that SP600125 can effetely inhibit the activity of JNK in human CCA cells. In order to determine the effects of JNK on human CCA cells proliferation and invasion, we treated QBC939, RBE and HCCC-9810 cells with various doses of SP600125 for indicated time periods. SP600125 inhibited the proliferation of human CCA cells in a dose- and time-dependent manner (Figure 1C). Furthermore, migration (Figure 1D) and invasion (Figure 1E) of human CCA cells were significantly suppressed by SP600125. These data indicate that aberrant activation of JNK signaling plays an important role in the pathogenesis of CCA.

**Figure 1:** JNK promotes human CCA cells proliferation and invasion. (A) Western blot analysis of phosphorylated JNK and phosphorylated c-Jun in human CCA cells. (B) SP600125 (SP) inhibits JNK activity in human CCA cells. After treated with various doses of SP600125 (SP) for 12 h, phosphorylated c-Jun in QBC939, RBE and HCCC-9810 cells was analyzed using western blot. (C) JNK blocking inhibits human CCA cells proliferation. QBC939, RBE and HCCC-9810 cells were treated with various doses of SP600125 (SP) for indicated time periods. Cell viability was determined by CCK8 assay. (D and E) JNK blocking suppresses human CCA cells migration and invasion. Human CCA cells were treated with SP600125 (SP, 20 µM) for 24 h before transferring to 24-well transwell chambers. The migration (D) and invasion (E) of QBC939, RBE and HCCC-9810 cells with or without SP600125 (SP, 20 µM) treatment were analyzed using transwell assay. Values are means±S.D. Columns, mean of three individual experiments; bars, SD. *Significantly different from control value.

### GRP78 promotes the proliferation and invasion of human CCA cells

To investigate the role of GRP78 in CCA, we tested the expression of GRP78 in human CCA cells. As shown in Figure 2A, QBC939, RBE and HCCC-9810 cells showed strong expression of GRP78. Tunicamycin-treated HepG2 cells were used as positive control. Given that both GRP78 induction and X-box binding protein 1 (XBP1) mRNA splicing are well-known biomarkers of the activation of unfolded protein response (UPR) [10], [11], [40], [41], spliced XBP1 mRNA was tested in human CCA cells. As shown in Figure 2B, the expression of spliced XBP1 mRNA was not detected in QBC939, RBE and HCCC-9810 cells. Tunicamycin-treated QBC939 cells were used as positive control. As the phosphorylation of eIF2α can induce GRP78 expression through activating transcription factor 4 (ATF4) independent of UPR elements [42], the eIF2α/ATF4 pathway was investigated in human CCA cells. Western blot analysis revealed strong expression of ATF4 and phosphorylated eIF2α in QBC939, RBE and HCCC-9810 cells (Figure 2C). The selective inhibitor of eIF2α phosphatase enzymes, salubrinal-treated HepG2 cells were used as positive control. Furthermore, ATF4 knockdown decreased the levels of GRP78 in human CCA cells (Figure 2D). Taken together, these results suggest that the eIF2α/ATF4 pathway, but not UPR, is responsible for the accumulation of GRP78 in human CCA cells.

**Figure 2:** eIF2α/ATF4 induces GRP78 accumulation in human CCA cells. (A) Western blot analysis of GRP78 in human cholangiocarcinoma cells. DMSO- and tunicamycin (Tun, 2.0 µg/ml)-treated HepG2 cells were used as negative and positive control, respectively. (B) RT-PCR analysis of spliced XBP1 mRNA in human CCA cells. Tunicamycin (Tun, 2.0 µg/ml)-treated QBC939 cells were used as positive control. (C) Western blot analysis of phosphorylated eIF2α and ATF4 in human CCA cells. Salubrinal (Sal, 25 µM)-treated HepG2 cells were used as positive control. (D) After transfected with ATF4 siRNA for 60 h, QBC939, RBE and HCCC-9810 cells were subjected to western blot analysis.

To confirm the tumorigenic role of GRP78 in human CCA cells, QBC939, RBE and HCCC-9810 cells were transfected with siGRP78 for indicated time periods. Compared with siGFP, siGRP78 inhibited the proliferation of human CCA cells in a time-dependent manner (Figure 3A). Furthermore, migration (Figure 3B) and invasion (Figure 3C) of QBC939, RBE and HCCC-9810 cells were significantly suppressed by GRP78 knockdown. The effects of siGRP78 on GRP78 suppression were confirmed by western blot (Figure 3D). Thus, GRP78 is a potent promoter of proliferation and invasion in human CCA cells.

**Figure 3:** GRP78 promotes human CCA cells proliferation and invasion. (A) GRP78 suppression inhibits human CCA cells proliferation. QBC939, RBE and HCCC-9810 cells were transfected with siGRP78 for indicated time periods. Cell viability was determined by CCK8 assay. (B and C) GRP78 suppression inhibits human CCA cells migration and invasion. To knockdown GRP78, human CCA cells were transfected with siGRP78 for 36 h before transferring to 24-well transwell chambers. The migration (B) and invasion (C) of QBC939, RBE and HCCC-9810 cells with or without siGRP78 treatment were analyzed using transwell assay. (D) The effects of siGRP78 on GRP78 suppression were measured using western blot. Values are means±S.D. Columns, mean of three individual experiments; bars, SD. *Significantly different from control value.

### JNK maintains high levels of GRP78 in human CCA cells

GRP78 has been previously shown to be induced by the JNK pathway through activator protein-1 (AP-1) upon lead treatment [43]. To investigate the association between JNK and GRP78, the effects of JNK inhibition on GRP78 accumulation were tested. It is notable that JNK inhibitor SP600125 treatment decreased the levels of GRP78 in a time-dependent manner in QBC939, RBE and HCCC-9810 cells (Figure 4A). Moreover, suppression the expression of JNK also decreased GRP78 accumulation in human CCA cells (Figure 4B). However, we found that AP-1 inhibitor curcumin had no demonstrable effects on GRP78 accumulation in human CCA cells (Figure S1), which indicating JNK regulates GRP78 independent of AP-1 in our study. To further confirm the role of JNK in regulating eIF2α-mediated GRP78 induction, HepG2 cells were used in our study. As shown in Figure 4C, SP600125 pretreatment inhibited eIF2α phosphatase enzymes inhibitor, salubrinal-induced GRP78 expression in HepG2 cells. These data indicate that JNK plays an important role in the accumulation of GRP78 upon the phosphorylation of eIF2α.

**Figure 4:** JNK maintains high levels of GRP78 in human CCA cells. (A) After treated with SP600125 (SP, 20 µM) for indicated time periods, GRP78 was analyzed using western blot in QBC939, RBE and HCCC-9810 cells. (B) After transfected with siJNK for 60 h, GRP78 was analyzed using western blot in QBC939, RBE and HCCC-9810 cells. (C) After treated with salubrinal (Sal, 25 µM) for 30 h with or without SP600125 (SP, 20 µM) preincubation for 1 h, GRP78 was analyzed using western blot in HepG2 cells. (D) After treated with tunicamycin (Tun, 2.0 µg/ml) for 24 h with or without SP600125 (SP, 20 µM) preincubation for 1 h, GRP78 was analyzed using western blot in HepG2 cells.

We addressed whether JNK participates in regulating the accumulation of GRP78 upon the activation of UPR. The levels of GRP78 were measured in HepG2 cells upon UPR inducer tunicamycin treatment. The data showed that JNK inhibitor SP600125 pretreatment had no demonstrable effects on tunicamycin-mediated GRP78 induction in HepG2 cells (Figure 4D). Taken together, these results suggest that JNK is involved in regulating eIF2α/ATF4-induced, but not UPR-induced GRP78 accumulation.

### JNK maintains high levels of GRP78 through the mTOR pathway in human CCA cells

It is known that the mTOR pathway, a crucial mediator of tumor progression, can be activated by JNK [44], [45], [46]. We therefore studied whether JNK regulates the mTOR pathway in human CCA cells. We found that JNK inhibitor SP600125 decreased the levels of phosphorylated ribosomal protein kinase S6 (p70S6K) (Figure 5A). Moreover, suppression of JNK expression also decreased the levels of phosphorylated p70S6K in human CCA cells (Figure 5B). As p70S6K is a downstream target of mTOR, we suggest that JNK has a crucial role in sustaining the activity of mTOR in human CCA cells. The mTOR pathway has been shown to be regulated by JNK through regulatory-associated protein of mTOR (Raptor) [45], [46]. To make sure whether JNK regulates mTOR signaling through Raptor in human CCA cells, the effects of JNK inhibition on the phosphorylation of mTOR and Raptor were investigated. The results showed that inhibition of JNK had no effects on the phosphorylation of mTOR in QBC939, RBE and HCCC-9810 cells (Figure 5C). Interestingly, JNK inhibitor SP600125 decreased the levels of phosphorylated Raptor in QBC939, RBE and HCCC-9810 cells (Figure 5D). As JNK inhibition decreased the phosphorylation levels of mTOR downstream targets, including p70S6K (Figure 5A) and eukaryotic translation initiation factor 4E-binding protein 1 (4E-BP1) (Figure 5D), it is reasonable to suggest that JNK regulates the activity of mTOR through Raptor in human CCA cells.

**Figure 5:** JNK promotes the activity of mTOR in human CCA cells. (A) After treated with SP600125 (SP, 20 µM) for indicated time periods, phosphorylated p70S6K in QBC939, RBE and HCCC-9810 cells was analyzed using western blot. Rapamycin (Rap, 20 nM)-treated cholangiocarcinoma cells were used as positive control. (B) After transfected with siJNK for 60 h, phosphorylated p70S6K in QBC939, RBE and HCCC-9810 cells was analyzed using western blot. (C) After treated with SP600125 (SP, 20 µM) for indicated time periods, phosphorylated mTOR in QBC939, RBE and HCCC-9810 cells was analyzed using western blot. (D) After treated with SP600125 (SP, 20 µM) for indicated time periods, phosphorylated Raptor and phosphorylated 4E-BP1 in QBC939, RBE and HCCC-9810 cells were analyzed using western blot.

We investigated whether mTOR participates in regulating the accumulation of GRP78 in human CCA cells. The levels of GRP78 were measured in mTOR inhibitor rapamycin-treated human CCA cells. Figure 6A showed that rapamycin decreased the levels of GRP78 in QBC939, RBE and HCCC-9810 cells in a time-dependent manner. Moreover, suppression the expression of mTOR also decreased the levels of GRP78 in QBC939, RBE and HCCC-9810 cells (Figure 6B). To further confirm the role of mTOR in regulating eIF2α-initiated GRP78 induction, HepG2 cells were treated with salubrinal with or without rapamycin preincubation. The data showed that rapamycin inhibited GRP78 induction upon salubrinal treatment (Figure 6C). It is notable that rapamycin had no demonstrable effects on tunicamycin-induced GRP78 expression in HepG2 cells (Figure 6D). These findings indicate that JNK suppresses eIF2α-initiated GRP78 induction through mTOR inhibition.

**Figure 6:** mTOR controls GRP78 synthesis in human cholangiocarcinoma cells. (A) After treated with rapamycin (Rap, 20 nM) for indicated time periods, GRP78 in QBC939, RBE and HCCC-9810 cells was analyzed using western blot. (B) After transfected with simTOR for 60 h, GRP78 in QBC939, RBE and HCCC-9810 cells was analyzed using western blot. (C) After treated with salubrinal (Sal, 25 µM) for 30 h with or without rapamycin (Rap, 20 nM) preincubation for 1 h, GRP78 was analyzed using western blot in HepG2 cells. (D) After treated with tunicamycin (Tun, 2.0 µg/ml) for 24 h with or without rapamycin (Rap, 20 nM) preincubation for 1 h, GRP78 in HepG2 cells was analyzed using western blot.

### JNK/mTOR regulates GRP78 induction through ATF4 in human CCA cells

Since ATF4 is required for GRP78 induction upon eIF2α phosphorylation [42], we tested the effect of JNK inhibition on the levels of ATF4 expression. As shown in Figure 7A, the levels of ATF4 were obviously decreased by JNK blocking in human CCA cells. However, JNK blocking had no effects on the phosphorylation of eIF2α (Figure 7A). Importantly, rapamycin treatment suppressed the expression of ATF4 without affecting the phosphorylation of eIF2α (Figure 7B). The data indicated that JNK/mTOR signaling regulates GRP78 induction through ATF4. To confirm the role of JNK/mTOR signaling in regulating ATF4 upon eIF2α phosphorylation, HepG2 cells were treated with salubrinal with or without SP600125 or rapamycin preincubation. The results confirm our hypothesis that JNK/mTOR signaling regulates ATF4 expression without affecting the phosphorylation of eIF2α (Figure 7C).

**Figure 7:** JNK/mTOR regulates GRP78 induction through ATF4 in human CCA cells. (A) After treated with SP600125 (SP, 20 µM) for 48 h, ATF4 and phosphorylated eIF2α in QBC939, RBE and HCCC-9810 cells were analyzed using western blot. (B) After treated with rapamycin (Rap, 20 nM) for 48 h, phosphorylated eIF2α and phosphorylated p70S6K in QBC939, RBE and HCCC-9810 cells were analyzed using western blot. (C) After treated with salubrinal (Sal, 25 µM) for 30 h with or without SP600125 (SP, 20 µM) and rapamycin (Rap, 20 nM) preincubation for 1 h, ATF4 and phosphorylated eIF2α were analyzed using western blot in HepG2 cells. (D) After treated with PF-4708671 (PF, 10 µM) and 4EGI-1 (50 µM) for 48 h, GRP78 and ATF4 in QBC939, RBE and HCCC-9810 cells were analyzed using western blot. (E) QBC939, RBE and HCCC-9810 cells were treated with rapamycin (Rap, 20 nM) for 12 h, and ATF4 and GRP78 mRNA levels were analyzed using real-time RT-PCR. Values are means±S.D. Columns, mean of three individual experiments; bars, SD. *Significantly different from control value.

Considering the role of mTOR signaling in controlling protein synthesis [47], [48], we investigated whether the mTOR pathway-controlled protein synthesis is required for ATF4 and GRP78 accumulation in human CCA cells. As shown in Figure 7D, eukaryotic translation initiation factor 4E/eukaryotic translation initiation factor 4G (eIF4E/eIF4G) interaction inhibitor 4EGI-1 decreased the protein levels of ATF4 and GRP78. It is notable that p70S6K inhibitor PF-4708671, which had no demonstrable effects on ATF4 and GRP78 accumulation, enhanced the decreasing of ATF4 and GRP78 in 4EGI-1-treated QBC939, RBE and HCCC-9810 cells (Figure 7D). Additionally, mTOR inhibition had no demonstrable effects on ATF4 mRNA levels (Figure 7E). Conversely, mTOR inhibition obviously decreased the mRNA levels of GRP78 (Figure 7E). These results indicate that mTOR controls eIF2α-initiated GRP78 induction through regulating ATF4 synthesis in human CCA cells.

As the PI3K/Akt pathway plays critical roles in regulating the activity of mTOR [49], we examined the effects of PI3K inhibition on eIF2α-induced ATF4 and GRP78 accumulation. As shown in Figure S2, PI3K inhibitor LY2940012 not only blocked the activity of mTOR but also inhibited the expression of ATF4 and GRP78 without affecting the phosphorylation of eIF2α in human CCA cells. These data support the notion that mTOR signaling is required for eIF2α-induced ATF4 and GRP78 accumulation.

### Expression of GRP78 and phosphorylated JNK in human CCA

To investigate whether JNK and GRP78 are involved in the progression of human cholangiocarcinoma, we examined the expression of GRP78 and phosphorylated JNK in human cholangiocarcinoma cases. As shown in Figure 8A, the expression of GRP78 and phosphorylated JNK was detected in human cholangiocarcinoma tissues, indicating that the JNK pathway and GRP78 are involved in the progression of human cholangiocarcinoma. Further studies are needed to investigate the association between JNK and GRP78 in human cholangiocarcinoma cases.

**Figure 8:** Expression of GRP78 and phosphorylated JNK in human CCA. (A) GRP78 and phosphorylated JNK in human CCA were analyzed using immunohistochemistry. (B) Summary of experimental findings. In human CCA cells, the phosphorylation of eIF2α initiates ATF4 expression, which then induces GRP78 accumulation. GRP78 plays an important role in promoting human CCA cells proliferation and invasion. Suppression of mTOR inhibits eIF2α-induced ATF4 expression, which leads to a decrease in GRP78 levels. JNK blocking decreases GRP78 levels through inhibiting the activity of mTOR. Similarly, PI3K/Akt blocking decreases GRP78 levels through inhibiting the activity of mTOR.

## Discussion

The inflammatory response pathways, including interleukin 6 (IL-6) and p38 MAPK pathways are implicated in the carcinogenesis and progression of CCA [7], [50], [51], [52], [53], [54]. However, the roles of the JNK pathway, another important pathway of inflammatory response [24], [32], [55], in CCA are remain unknown. The present work reveals that GRP78 contributes to the oncogenic action of JNK in human CCA cells.

GRP78 has been reported to be associated with a wide variety of human malignancies, such as prostate, liver and breast cancer [15], [17], [40], [56], [57], [58], [59]. However, it is unknown whether GRP78 is involved in the progression of CCA. Importantly, both human CCA cells and CCA tissues showed strong expression of GRP78. Based on the data that suppression GRP78 by siRNA inhibited the proliferation and invasion of human CCA cells, we suggest GRP78 exerts pro-tumorigenic action in human CCA. As the accumulation of GRP78 is a classic indicator of the onset of UPR [10], [11], it is interesting to investigate whether GRP78 accumulation is caused by UPR in human CCA cells. As the splicing of XBP1 mRNA, another well-known biomarker of UPR [41], can't be detected in human CCA cells, it's reasonable to suggest that the accumulation of GRP78 is not caused by UPR in human CCA cells. Interestingly, human CCA cells showed high levels of phosphorlated eIF2α and its downstream target ATF4. Because the eIF2α/ATF4 pathway can induce GRP78 expression without the onset of UPR [42], it is reasonable to suggest that eIF2α/ATF4 signaling is responsible for the accumulation of GRP78 in human CCA cells. This speculation is supported by our data which demonstrated that ATF4 knockdown obviously decreased the accumulation of GRP78 in human CCA cells.

Our data show that both human CCA cells and CCA tissues display strong activity of JNK. Based on the data that blocking JNK by SP600125 inhibited the proliferation and invasion of human CCA cells, we suggest that JNK promotes the carcinogenesis and progression of CCA. An important question now before us is how JNK exerts its oncogenic potential in human CCA cells. Our data showed that blocking the activity or suppression the expression of JNK obviously decreased the levels of GRP78 in human CCA cells. As our data demonstrated that GRP78 is involved in the progression of human CCA, it is reasonable to suggest that JNK exerts its pro-tumorigenic effects, at least in part, through GRP78 signaling. Considering the accumulation of GRP78 is eIF2α/ATF4-dependent in human CCA cells, we investigated the role of JNK in regulating the specific inhibitor of eIF2α phosphatase enzymes salubrinal-mediated GRP78 induction in HepG2 cells. As expect, JNK inhibition decreased the induction of GRP78 in HepG2 cells upon salubrinal treatment. However, JNK inhibition had no demonstrable effects on UPR-mediated GRP78 induction in HepG2 cells. Thus, JNK signaling regulates eIF2α/ATF4-initiated GRP78 accumulation, but not UPR-induced GRP78 expression.

In order to uncover the detailed mechanism of JNK in regulating GRP78 accumulation, we investigated the effects of JNK inhibition on the eIF2α/ATF4 pathway. Based on our findings, we proposed that JNK regulates ATF4 expression without affecting the phosphorylation of eIF2α in human CCA cells. Considering the mTOR pathway, which can be regulated by JNK, plays a pivotal role in protein synthesis [47], [48], we suspected that JNK might decrease eIF2α-induced ATF4 and GRP78 expression through the mTOR pathway. This hypothesis was supported by the data that JNK inhibition decreased the activity of mTOR, and mTOR inhibition suppressed eIF2α-initiated ATF4 and GRP78 induction. In agreement with previous reports [45], [46], we found that JNK promoted the activation of mTOR signaling through Raptor. It is notable that mTOR inhibition decreased the induction of ATF4 and GRP78 in HepG2 cells upon salubrinal treatment. However, mTOR inhibition had no demonstrable effects on UPR-initiated GRP78 induction in HepG2 cells. Thus, mTOR signaling is required for eIF2α-initiated GRP78 accumulation, but is not required for UPR-induced GRP78 expression. The detailed mechanism for this difference is not clear and needs further research. As p70S6K and 4E-BP1, two downstream targets of mTOR, are responsible for mTOR-controled protein synthesis, we focused on the role of p70S6K and 4E-BP1 in eIF2α-initiated ATF4 and GRP78 induction. Inhibiting eIF4E/eIF4G interaction substantially decreased ATF4 and GRP78 accumulation. The inhibitor of p70S6K alone had no appreciable effects on ATF4 and GRP78 accumulation, but the synergistic effect of p70S6K inhibition on eIF4E/eIF4G interaction inhibition-mediated ATF4 and GRP78 down-regulation was observed. Our data suggest that JNK contributes to ATF4 and GRP78 accumulation through regulating mTOR-mediated ATF4 synthesis. This notion is supported by the data that mTOR inhibition suppressed ATF4 expression without affecting its mRNA levels. The role of mTOR in regulating the eIF2α/ATF4/GRP78 pathway was further supported by the finding that the PI3K/Akt blocking-mediated mTOR inhibition suppressed ATF4 and GRP78 expression upon eIF2α phosphorylation.

In conclusion, we found that GRP78 contributes to the pro-tumorigenic function of JNK in human CCA cells. High levels of phosphorylated JNK and GRP78 are found in human CCA cells and CCA tissues. Both JNK and GRP78 have a vital function in promoting the proliferation and invasion of human CCA cells. JNK sustains high levels of GRP78 through mTOR/p70S6K/4E-BP1 signaling in human CCA cells (Figure 8B). More detailed studies on the mechanism of JNK aberrant activation and GRP78 aberrant accumulation in CCA will contribute to the understanding of molecular mechanism of cholangiocarcinogenesis and the development of new therapeutic strategies against CCA.

## Supporting Information

Figure S1 AP-1 has no effects on eIF2α-initiated GRP78 accumulation in human CCA cells. After treated with AP-1 inhibitor curcumin (25 µM) for 48 h, GRP78 in QBC939, RBE and HCCC-9810 cells was analyzed using western blot.
(TIF)

Figure S2 PI3K/Akt blocking-mediated mTOR inhibition suppresses ATF4 and GRP78 expression in human CCA cells. After treated with LY294002 (LY, 20 µM) for 48 h, GRP78, ATF4 and phosphorylated eIF2α in QBC939, RBE and HCCC-9810 cells were analyzed using western blot.
(TIF)
